# An analysis of changes in the prevalence and patterns of intimate partner violence against women in seven Asian countries

**DOI:** 10.1186/s12905-023-02534-6

**Published:** 2023-07-31

**Authors:** Seema Vyas, Henrica A.F.M Jansen, Jessica Gardner, Sujata Tuladhar, Kate Hammond, Kristin Diemer

**Affiliations:** 1 Independent researcher, London, United Kingdom; 2 Independent researcher, Bangkok, Thailand; 3 UNFPA Asia-Pacific Region, Bangkok, Thailand; 4 University of Melbourne, Melbourne, Australia

**Keywords:** Intimate partner violence, South Asia, Southeast Asia, Domestic violence

## Abstract

**Background:**

Assessments of changes in prevalence and patterns of violence against women are critical to inform prevention and response approaches and to monitor progress towards elimination. Most countries in the Asia Region have data on violence and several have completed second and third waves of surveys. This study sought to assess and compare the prevalence and patterns of physical and/or sexual partner violence in seven Asian countries with at least two rounds of comparable national-level data.

**Methods:**

We conducted primary descriptive analyses using Demographic and Health data from India, Nepal, and Pakistan (South Asia), and from Cambodia, the Philippines, Timor-Leste, and extracted data from reports from Vietnam (Southeast Asia). We examined differences in partner violence by type of violence, reference periods, severity of violence, and age group. Pearson chi-square tests and Mantel-Haenszel test for trend were used to assess whether differences between time points were significant (p < 0.05).

**Results:**

Prevalence and patterns of violence vary across countries and sub-regions. In Southeast Asia, women in Cambodia and Vietnam experienced increasing and relatively high levels of sexual violence alongside declining physical violence. Reported levels of violence were lowest in the Philippines and prevalence showed consistent declines. Timor-Leste stands out as having the highest prevalence of physical partner violence, and there were consistently significant increases in estimates. Women in South Asia experienced predominantly physical violence and there were consistent declines in all three countries, though physical violence increased among older women in India.

**Conclusions:**

Data from Asian countries where more than one prevalence survey had been done provided a unique opportunity to analyse differences in estimates of violence against women at two time points. Deeper analyses into types and severity of violence revealed that overall prevalence estimates hid more complex patterns. There are clear limitations in using survey data to understand the nuances which highlighted the need for depth analysis identifying contextual factors of violence to inform situation specific policies and interventions for the greatest impact. It is also clear that more than two data points are necessary to identify change over time, and interventions driving or preventing that change.

## Introduction

Violence against women is a human rights violation that harms women and communities, and burdens countries around the world [1, 2]. Intimate partner violence is one of the most common forms of violence against women, and estimates reveal that globally, 26% of ever-partnered women have experienced physical and/or sexual partner violence by an intimate partner in their lifetime [2]. Such violence, moreover, is associated with serious physical, mental and sexual and reproductive health risks to women and their families [3, 4]. and negatively impacts on women’s workforce productivity and household economies [5]. The pervasiveness and widespread consequences of violence has resulted in a call for a comprehensive response across the globe.

Spurred by the urgent need for action, the United Nations General Assembly set Sustainable Development Goal (SDG) target 5.2—to eliminate all forms of violence against all women and girls [6]. This has put renewed emphasis on violence prevention and response approaches, with countries being encouraged to monitor change in prevalence over time using quantifiable indicators such as those measuring intimate partner violence. To date, much of these data have come from either dedicated violence against women surveys which use established safe and ethical methodologies (such as that developed for the World Health Organization’s Multi-country Study on Women’s Health and Domestic Violence against Women, hereafter `referred to as WHO-methodology), or from Demographic and Health Surveys (DHS) that include the DHS domestic violence module.

In the Asia Region, out of 19 countries with data on violence against women, eight have completed second and third waves of national prevalence surveys using comparable methods [7]. This study assesses changes in prevalence of physical and/or sexual violence by intimate partners over time in seven of these countries where either the data or reports were publicly available: India, Nepal and Pakistan (in South Asia) and Cambodia, Philippines, Timor-Leste and Vietnam (in Southeast Asia). Further, this study explores differences in the levels and patterns of the underlying types of violence, both between countries, as well as and between the two Asia sub-regions. Data or reports from Bangladesh were not publicly available and therefore, this study does not assess changes in that country.

## Methods

### Survey methodology

Data for this study comes from nationally representative DHS and WHO-methodology based prevalence surveys. The WHO-methodology was put into practice through the WHO Multi-country Study on Women’s Health and Domestic Violence against Women, first published in 2005 [8]. A primary impetus for this study and the development of a new methodology was the existing inconsistencies in how intimate partner violence data was collected across time periods and in different settings [8]. The WHO methodology aimed to create consistency in measuring prevalence estimates on partner violence for the purpose of comparison or to understand differences and changes in the extents, patterns, and factors associated with violence across time periods and in different cultural settings [8]. The methodology developed for the WHO Multi-country study is now seen as best practice when conducting population-based studies of violence against women [9], and this methodology has been replicated or adapted in over 20 countries in the Asia-Pacific region, and many more countries around the world [7].

While WHO-methodology based studies are dedicated surveys specifically designed to gather detailed information on different types of violence against women, the DHS are large national sample surveys that are designed to measure demographic and health trends in the population [8, 10]. The DHS is typically conducted every five years in a country through a questionnaire administered to all women aged 15–49 in a household. Questions cover a range of topics including women’s reproductive and sexual health, and knowledge about HIV. Increasingly, DHS have included a standardised module on domestic violence which, in line with the WHO’s ethical guidelines [8, 11], is administered to one randomly selected eligible woman in a household.

Early administration of surveys based on the WHO methodology randomly selected one woman aged 15–49 per household to be invited for interview [12]. More recently, in the Asia Region the age range has increased to now include older women up to age 64 or older. A second distinction between DHS and WHO-methodology based surveys is that the DHS typically administers questions on partner violence to women who have ever been married or who have ever lived with a male partner [13], while some surveys using the WHO-methodology include women and girls in dating relationships. A third distinction is that WHO-methodology based surveys ask women about their experiences from any partner (current or former) [12], while in all DHS, respondents are asked whether their current partner (asked to married or cohabiting women) or most recent partner (asked to widowed, divorced or separated women) perpetrated any of the acts of violence [13]. More recent DHS ask an additional question whether any of the acts were perpetrated by a previous/former partner.

Because we explore differences and changes over time, we focussed our analyses on the seven Asian countries where either DHS or the WHO-methodology based surveys had been applied over two or more different time points. For these countries, we conducted our analyses using data from a total of seventeen surveys spanning from 2000 to 2019; fifteen surveys were DHS and two surveys were based on the WHO methodology (Table 1). The number of ever partnered women answering questions on domestic violence ranged from 2,162 (Timor-Leste 2009–2010) to 69,484 (India 2005–2006).

It is important to note that a minimum of three time points is required for trend analysis [14], as two time points are not conclusive of trends. Due to this study including countries with either two or three time points, our data should therefore be interpreted as changes rather than trends.

### Measure of partner violence against women

Both DHS and WHO methodologies ask behaviourally specific questions on women’s experiences of acts of violence perpetrated by their partner. The questions that we use for this analysis focus on physically violent acts —which start off moderate in severity such as being pushed or slapped, through to severe violence such as having a knife or other weapon used against them — and on acts of sexual violence. The questions asked in each survey and of relevance for this analysis are detailed in Box 1.

**Table:** 

Box 1: Survey questions on domestic violence against women	
DHS	WHO
**Physical violence**	**Physical violence**
Pushed, shaken or thrown something	Slapped or thrown something that could hurt
Slapped	Pushed, shoved, or pulled hair
Twisted arm or pulled hair	
***Severe physical violence***	***Severe physical violence***
Punched or hit with something that could hurt	Hit with his fist or with something else that could hurt
Kicked, dragged or beaten up	Kicked, dragged, or beaten up
Choked or burnt on purpose	Choked or burnt on purpose
Threatened or attacked with a knife, gun or other weapon	Threatened to use or actually used a gun, knife or other weapon
**Sexual violence**	**Sexual violence**
Physically forced to have sexual intercourse	Forced to have sexual intercourse
Forced to perform any other sexual acts	Had sexual intercourse because afraid of what partner might do
Tried to or attempted to force to have sexual intercourse or perform any other sexual act^a^	Forced to do something sexual that was degrading or humiliating
Persuaded or threatened to have sexual intercourse or perform other sexual acts^b^	Forced to have sex with another person^c^

^a^ Included in Philippines 2008 & 2013

^b^ Included in India 2015-16, Nepal 2016-17, Pakistan 2017-18, Cambodia 2014, Philippines all 3 survey rounds, Timor-Leste 2016

^c^ Included in Vietnam 2010

The questions asked about acts of physical violence were consistent across survey rounds and within each country. Acts to measure sexual violence varied slightly. For example, an additional question *forced with threats to have sexual intercourse or perform other sexual acts* was included in more recent DHS. In Vietnam, which used the WHO methodology, the act *forced* [by an intimate partner] *to have sex with another person* was an adaptation included only in the 2010 survey, and because it did not yield many additional cases was not included in the 2019 survey [15, 16]. Despite these slight differences, for each survey we included all questions that were asked to measure sexual violence. Lifetime physical and/or sexual partner violence was identified if a woman indicated she had “ever” experienced one or more acts of physical or sexual violence. Current partner violence was identified if a woman indicated any of these acts occurred in the past 12 months.

### Analysis

For each Asian country with multiple DHS we requested access to the datasets, which was reviewed and granted by the DHS programme, and carried out primary analysis. For the Viet Nam WHO-methodology based surveys, secondary analyses from findings published in reports were conducted.

We examined the prevalence of physical and/or sexual partner violence by reference period (lifetime, current) by type of violence (physical, sexual) and by severity of physical violence (moderate, severe). Pearson chi-square test and Mantel-Haenszel test for change (where there are three data points) were performed to assess significant differences or changes in these parameters. We also examined differences in the prevalence of partner violence by age group and compared these changes by survey timeframe.

All data in the DHS applied weights and standard errors were adjusted for the surveys multi-stage cluster design. In Pakistan, the 2012–2013 DHS only asked questions about acts of physical violence, and therefore, we only compare prevalence of physical partner violence over time. Moreover, the 2012–2013 survey did not include respondents from the area of Azad Kashmir, and the 2017–2018 DHS calculated separate weights for the Gilgit Baltistan Region, and therefore, both areas are excluded from the analysis.

Verbal informed consent was obtained from all individual respondents included in all original surveys. This study only analyses publicly available data gathered as part of the DHS programme and from WHO reports; therefore, we did not seek additional ethical approval for this study.

## Results

The socio-demographic characteristics of ever-partnered women, who answered questions on violence, are shown in Table 1. In the six countries which used the DHS methodology, across all survey rounds, the mean age of respondents (aged 15–49) ranged from 31.6 years in Nepal (2011) to 34.7 years in the Philippines (2017).

The average age of first marriage or cohabitation was earlier in all South Asian countries—range 17.1 years in India (2006) to 19.4 years in Pakistan (2018)—, than in Southeast Asia—range 19.5 years in Cambodia (2000) to 21.3 years in the Philippines (2008). In all countries, with the exception of the Philippines, the average age at first marriage or cohabitation increased slightly over time; in the Philippines, average age remained stable across the three survey rounds. The vast majority of surveyed women, over 85% in each study, was either married or cohabiting (unmarried and living with their male partner) at the time of interview. In South Asian countries, approximately 95% of women were married, cohabiting relationships were not captured in the India and Pakistan surveys and virtually no women were in a cohabiting relationship in Nepal. The partnership status of women in the four Southeast Asian countries was more varied. In Cambodia and Vietnam proportionately few women were cohabiting, however, a notable trend in the Philippines and in Timor-Leste is the increase in women reporting that they were living with their partner and unmarried—27.3% in the Philippines in 2017 (up from 17.1% to 2008) and 12.5% in Timor-Leste in 2016 (up from 3.9% in 2009-10).

The percentage of women who had at least secondary education increased over time in each country, except in Vietnam where educational attainment slightly declined and may be explained by the widened age range of respondents for the second survey. Variability in educational attainment was greater across the Southeast Asian countries where the percentage with at least secondary education ranged from a low of 12.7% (Cambodia 2000) to a high of 81.5% (Philippines 2017). In South Asian countries, levels of secondary education were similar in the first time point and increased over time, with a more dramatic increase, albeit spanning over a longer time frame, being found in India (36.6% in 2005–2006 to 57.5% in 2019–2021).

**Table 1:** Survey characteristics and respondent demographics (ever-partnered women interviewed with the domestic violence module)

Country	Year	Number ever partnered women	Mean age *(S.E)*	Mean age at 1st marriage cohabitation *(S.E)*	Married (%)	Live together (%)	Widowed (%)	Separated / divorced (%)	No education (%)	Primary (%)	Secondary or more (%)
*South Asia*											
India*	2005-06	69,484	31.66 *(0.06)*	17.13 *(0.03)*	94.0	–	4.0	2.0	48.1	15.4	36.6
	2015-16	66,013	33.17 *(0.06)*	18.41 *(0.03)*	94.5	–	4.0	1.5	32.5	14.3	53.2
	2019-21	63,815	34.22 *(0.07)*	18.47 *(0.04)*	94.0	–	4.3	1.7	28.6	13.9	57.5
Nepal	2011	3,505	31.56 *(0.23)*	17.38 *(0.11)*	95.7	–	3.1	1.3	48.8	18.2	33.0
	2016-17	3,826	32.08 *(0.19)*	17.65 *(0.09)*	96.7	0.0	2.2	1.0	41.9	18.7	39.4
Pakistan**	2012-13	3354	32.84 *(0.23)*	18.95 *(0.13)*	95.4	–	3.4	1.1	57.5	15.6	26.9
	2017-18	3303	32.13 *(0.22)*	19.44 *(0.12)*	96.7	–	2.4	0.9	49.6	15.5	34.9
*Southeast Asia*											
Cambodia	2000	2,403	34.32 *(0.25)*	19.50 *(0.09)*	86.5	–	9.1	4.5	31.0	56.3	12.7
	2005-06	2,294	34.17 *(0.26)*	19.60 *(0.12)*	87.9	0.4	5.3	6.4	25.2	58.6	16.2
	2014	3,499	33.46 *(0.26)*	20.00 *(0.09)*	90.2	1.5	3.5	4.8	15.3	53.2	31.6
Philippines	2008	7,157	33.84 *(0.11)*	21.27 *(0.07)*	77.0	17.1	2.1	3.8	1.5	23.3	75.2
	2013	8,160	34.52 *(0.12)*	21.17 *(0.07)*	70.1	21.9	2.1	6.0	1.6	20.7	77.8
	2017	13,215	34.67 *(0.14)*	21.20 *(0.08)*	65.9	27.3	1.8	4.9	0.9	17.6	81.5
Timor-Leste	2009-10	2,162	33.54 *(0.25)*	19.97 *(0.13)*	90.2	3.9	3.5	2.4	38.5	25.3	36.3
	2016	3,694	33.30 *(0.18)*	20.46 *(0.10)*	83.7	12.5	1.8	2.0	29.0	18.7	52.4
Vietnam***	2009-10	4,562	–	–	89.8	0.2	5.2	4.5	9.0	26.0	65.0
	2018-19	5,553	–	–	86.9	0.2	5.3	4.8	16.9	22.7	60.4

* Age at 1st marriage/live together unmarried not asked to widowed, separated or divorced women in 2015–2016 survey–mean age calculated among currently married women

** Analyses excludes Azad Kashmir and Gilgit Baltistan

*** Ever-partnered includes women who have been in dating relationships only; respondent mean age and age at 1st marriage not documented in reports

*S.E. Standard error*

### Prevalence of partner violence over survey time points

Table 2 presents estimates on the prevalence of lifetime and current physical and/or sexual partner violence for each country and by survey time point. By sub-regions, there was greater variation in the prevalence and patterns of partner violence in Southeast Asian countries compared with South Asian countries.

In the South Asian countries, the prevalence of lifetime and current physical and/or sexual partner violence were highest in India. The prevalence of lifetime and current physical and/or sexual violence in Nepal and Pakistan (data available for the second time point only in Pakistan) were more similar. In the first time point, prevalence measured 28.2% in Nepal and 37.2% in India, and there were significant declines in violence (p < 0.001) in both countries where, by the most recent time point, prevalence measured 24.3% in Nepal and 29.1% in India. Current violence measured 14.3% in Nepal and 23.0% in India in the first time point, and when changes were assessed statistically, a notable difference to emerge between the two countries was that current violence significantly declined in Nepal (p < 0.001) but significantly increased to 24.0% in India (p < 0.001). The increase in prevalence of current violence in India and the higher ratio of current to lifetime violence over subsequent time points, compared to the first time point, suggests that violence continued, once it had started, for more women.

Across the Southeast Asian countries and in the first time point, the prevalence of lifetime physical and/or sexual partner violence were similarly lower in Cambodia and in the Philippines (17.1% and 17.3% respectively) and similarly higher in Vietnam and in Timor-Leste (34.4% and 34.2% respectively). There was a significant decreasing change in the prevalence of violence in the Philippines (p < 0.001 lifetime and current), and in the prevalence of current partner violence in Cambodia (p < 0.001), but there was, however, no significant change association in the prevalence of lifetime partner violence (p = 0.107). In both countries there were steady decreases across time points in the prevalence of current violence relative to lifetime violence, highlighting that violence had ceased (at least temporarily) for proportionately more women.

In Timor-Leste, prevalence of violence significantly increased over the two time points (p < 0.004 lifetime; p < 0.001 current). Furthermore, the estimates of current violence were almost as high as lifetime violence, and in both time points, depicting that the vast majority of women consistently continued to live with violence once it had started. In Vietnam, lifetime violence declined from 34.4% in the first time point to 32.0% in the second, a result that was statistically significant (p < 0.001), however, prevalence of current violence remained static (p = 0.857). In both time points, reported experiences of current violence were much lower than lifetime violence, depicting that violence had ceased (at least temporarily) for the majority of women who had ever experienced violence, and this level of violence cessation was fairly stable over the two time points.

**Table 2:** Prevalence of lifetime and current partner violence

		% Physical and/or sexual partner violence				% Physical partner violence				% Sexual partner violence			
Country	Study year	Lifetime	p-value	Current	p-value	Lifetime	p-value	Current	p-value	Lifetime	p-value	Current	p-value
*South Asia*													
India	2006	37.2	< 0.001	23.0	< 0.001	35.1	< 0.001	20.5	< 0.001	10.8	< 0.001	7.0	< 0.001
India	2016	30.9		23.9		29.8		22.5		7.0		5.7	
India	2021	29.1		24.0		28.3		23.0		6.1		5.2	
Nepal	2011	28.2	< 0.001	14.3	< 0.001	23.1	0.76	10.7	0.325	14.3	< 0.001	7.7	< 0.001
Nepal	2017	24.3		11.2		22.8		10.0		7.0		4.0	
Pakistan*	2013					27.0	< 0.001	18.0	< 0.001	n.a		n.a.	
Pakistan*	2018	23.7		14.5		22.9		13.6		4.8		3.6	
*Southeast Asia*													
Cambodia	2000	17.1	0.107	15.2	< 0.001	16.4	0.02	14.6	< 0.001	3.6	< 0.001	3.2	0.035
Cambodia	2006	13.7		9.0		12.8		8.3		2.7		1.7	
Cambodia	2014	18.2		10.9		16.2		9.3		5.5		3.9	
Philippines	2008	17.3	< 0.001	10.0	< 0.001	14.4	< 0.001	7.3	< 0.001	7.0	< 0.001	4.8	< 0.001
Philippines	2013	14.7		7.1		12.7		5.3		5.9		3.3	
Philippines	2017	12.2		5.4		11.0		4.3		4.0		2.2	
Timor-Leste	2010	34.3	0.004	30.4	< 0.001	33.5	0.017	29.6	0.006	2.3	< 0.001	2.0	< 0.001
Timor-Leste	2016	38.1		34.6		36.6		33.1		5.0		4.8	
Vietnam**	2010	34.4	0.011	9.0	0.857	31.4	< 0.001	6.4	< 0.001	9.9	< 0.001	4.2	< 0.001
Vietnam**	2019	32.0		8.9		26.1		4.6		13.3		5.7	

* Physical violence only, excludes Azad Kashmir and Gilit Baltistan

** Violence from any partner

n.a.= not available (in Pakistan data on sexual violence were not collected in 2012–2013)

p-values were calculated using Pearson chi-square (Mantel-Haenszel test for trend in Cambodia, India, and the Philippines) to test, for each country, if the values in the time series indicate a change, with smaller p-value indicating a larger likelihood of a difference between time points.

Exploring changes by type of violence provides information on what type of violence contributed to the measured differences in prevalence across countries. In all countries from both sub-regions, the dominant type of violence women experienced was physical.

In all three countries in South Asia, the prevalence of physical partner violence measured almost as high as the prevalence of overall violence. There were different patterns in how estimates of physical partner violence varied over time across the countries. In Nepal there were no significant differences in the reported level of either lifetime or current physical violence over the two time points. In India, lifetime physical violence significantly declined across the three time points, however, current physical violence significantly increased across the three time points (p < 0.001). In Pakistan both lifetime and current physical partner violence significantly declined (p < 0.001). The prevalence of lifetime sexual partner violence measured 14.3% in Nepal and 10.8% in India, a level which had significantly declined (p < 0.001) by the most recent time point to 7.0% in Nepal and to 6.1% in India. The prevalence of current sexual partner violence also significantly declined (p < 0.001) over time in both countries. The prevalence of reported sexual partner violence was lowest in Pakistan and measured 4.8% (lifetime) and 3.6% (current).

Physical violence was also the dominant type of violence women experienced in Southeast Asia, and particularly so in Timor-Leste where prevalence was almost as high as overall violence; in contrast, the prevalence of sexual violence in Timor-Leste was among the lowest in the sub-region. Furthermore, in Timor-Leste, estimates of physical partner violence significantly increased over the time points (p < 0.001 lifetime and current). This is in contrast to the significant decrease in both lifetime and current physical partner violence in Cambodia, the Philippines, and Vietnam over the time points. While the prevalence of sexual violence significantly declined in the Philippines, there were significant increases in reported rates of sexual violence in Timor-Leste (p < 0.001), Vietnam (p < 0.001) and Cambodia (lifetime p < 0.001; current p = 0.035).

### Overlap in type of violence

Figure 1a and b show prevalence of partner violence broken down by whether women had experienced only physical violence, both physical and sexual violence, and only sexual violence in their lifetime (Fig. 1a) and in the past 12 months (Fig. 1b).

In India and Pakistan, the majority of cases of lifetime and current violence involved only physical violence, and women who experienced sexual violence mostly experienced it in combination with physical violence. By contrast, in Nepal and in the first time point approximately one half of women experienced sexual violence either in combination with physical violence or only sexual violence. In both India and Nepal, the prevalence of sexual violence, either in combination with physical violence or sexual only violence, had fallen between the first and last reference points. The prevalence of current physical only violence however, increased in both countries over the same periods. These findings confirm that in India physical violence drives the higher prevalence of overall current violence, and that in Nepal declines in sexual violence drives the overall decline.

In Southeast Asia, with the exception of Vietnam, the majority of women who experienced violence experienced physical only violence. In Vietnam, the proportion of women who experienced sexual violence, and in particular sexual only, increased over the time points to become the dominant type of current violence by the second time point. For example, lifetime prevalence of sexual only violence increased from 3.0% in the first time point to 5.9% in the second time point, and these figures were 2.6% and 4.3% respectively when considering current levels. This implies that by the second time point almost one in five cases of lifetime violence was sexual only and almost one half of cases in the past 12 months were sexual only. In the Philippines, there were declines in all three measures of partner violence and for both reference periods. By contrast, all three measures of partner violence increased in Timor-Leste, although the vast majority of women continued to experience physical only violence. In Cambodia, like Vietnam, the prevalence of sexual only violence generally increased over time and for both reference periods. While current physical only violence declined over time, there was no other clear change in the estimates of lifetime physical only violence or in the prevalence of lifetime or current physical and sexual violence.

**Fig. 1:** Percent ever-partnered women who experienced physical only violence, physical and sexual violence, or sexual only violence in (**a**) their lifetime (**b**) the last 12 months

### Severity of physical partner violence

Physical violence was categorised as moderate only and severe depending on the act of violence (Box 1). In South Asia, the proportion of women who experienced severe physical violence in their lifetime declined in each country across time points i.e., from 10.7 to 8.7% (Pakistan); 15.1–11.9% to 11.3% (India); and 12.0–11.6% (Nepal) (Fig. 2a). Current levels also declined in Nepal and Pakistan but increased in India from 8.5% in the first time point to 9.5% by the third time point (Fig. 2b).

**Fig. 2:** Percent ever-partnered women who experienced moderate only physical violence or severe physical violence in (**a**) their lifetime (**b**) the last 12 months (percent for Vietnam in past 12 months is all physical violence)

In Southeast Asia, both lifetime and current estimates of severe physical violence declined in the Philippines across the three time points. In Timor-Leste, both lifetime and current severe physical violence increased over time, and additionally, the proportion of women who experienced severe physical violence, as a proportion of any physical violence, increased over time. In Cambodia and Vietnam, there was no notable difference in the proportion of women who experienced severe physical violence in their lifetime or in the past 12 months (Cambodia) between the first and last time points —severity of current violence in Vietnam could not be assessed.

### Changes in physical and/or sexual partner violence by age group

Age specific patterns of physical and/or sexual partner violence over time are shown for each country in Fig. 3. In all three countries in South Asia, data suggest that lifetime partner violence declined over time in all age groups, except for a slight increase among 15–19-year-olds in Nepal. The differences in the levels of current violence, however, contrasted by country; in Pakistan, current (physical) violence declined over time in each age group, violence increased in the youngest age group in Nepal and increased in the oldest age groups in India.

In the Philippines, declines in lifetime and current partner violence were observed across all age groups, except current violence among the youngest women increased slightly between 2013 and 2017. In Timor-Leste, increases in lifetime and current partner violence were observed in all age groups. In Vietnam, with the exception of the 18–24 age group, which saw a notable decline in current violence, there was no notable change in prevalence across the other age groups. The changes in violence by age group in Cambodia showed no apparent consistent pattern.

**Fig. 3:** Percent physical and/or sexual partner violence in lifetime and past 12 months (current) by age group

## Discussion

In this study we explore evidence on the differences and changes in the prevalence and patterns of physical and/or sexual partner violence in seven Asian countries where two or more nationally representative surveys with comparable methods have been conducted. Before assessing the implications of our findings, an important limitation of this study to highlight is that two time points are not conclusive of trends [14], and we suggest a minimum of three time points for trend analysis. Due to four out of the seven countries in this study not having comparable IPV prevalence data across three or more time points, we are as yet unable to identify whether changes over time are indicative of larger trends in those countries. Because national violence against women prevalence surveys are highly complex, sensitive and resource intensive, they should only be conducted with five to ten year intervals, therefore additional data points will not be soon available. The current investigation of highly comparable data from as many as seventeen surveys in seven countries does enable exploring whether the situation on violence against women appears to be changing. These changes, when tested, yielded significant results, likely due to the large sample sizes of DHS data.

The data from our study has shown that measures of prevalence by type of violence and patterns of violence vary across countries and the sub-regions. That there are contrasting changes in the prevalence of violence is consistent with findings from other regions including a recent study which reviewed data from the Americas. The latter study also found decreases in certain types of partner violence in some countries, while in other countries prevalence did not differ at all or increased [16].

Among the main findings in this study is that women in Southeast Asia appear to have a more diverse experience of violence than women in South Asia. In Cambodia and Vietnam, women experience increasing and relatively high levels of sexual violence in a context where there is evidence of some significant declines in physical partner violence from one time point to the next. It is unclear, however, whether these increases in reported sexual violence reflect actual increases in violence or are the result of social change and that women are more open to disclosing their experiences. Women in the Philippines have the lowest reported levels of violence across all the countries and the measure of prevalence showed consistent declines for both types of violence and for the severity of physical violence and over both the lifetime and current reference periods.

The pattern of violence in Timor-Leste, however, was very different to that in the other Southeast Asian countries. It is the country with the highest prevalence of partner violence and there are consistent and significant increases in this prevalence from the first to the second time point. Furthermore, unlike in Cambodia and Vietnam, women’s experiences of violence in Timor-Leste are ongoing and almost exclusively physical. This finding in Timor-Leste is worrisome if the implication is that women are experiencing violence on an ongoing basis because they have few response options including to leave an abusive relationship. This highlights the urgent need for the implementation and/or scale-up of prevention and essential response services.

In South Asia, women’s experiences of violence are predominantly physical. There was a fairly consistent decline in the levels of lifetime and current violence (mostly sexual violence in India and Nepal) in the respective time points included for each country. The notable exception was the increasing trend in current physical violence in India which, in the context of declining lifetime physical violence, suggests that over the fifteen or so years the three studies were conducted, while fewer women overall reported that they had experienced violence in their lifetime, for proportionately more women the violence had continued.

Exactly what drives these changes in partner violence is an open question. An intuitive conclusion is that these are the result of a “cohort effect”, that is, they are driven by experiences among younger women and possibly because of demographic shifts such as increasing age at marriage/cohabitation and improvements in educational attainment. Evidence from low- and middle-income countries has documented that the protective benefits of education are generally realised with at least secondary schooling [16–19]. However, there may be other social, political, and environmental factors that impact prevalence of IPV at any given time. Previous studies using WHO and DHS data have showed that political insecurity and upheaval, conflict, and natural disasters all correlate with an increase in levels of IPV [19–23], all or some of which may be relevant when measuring IPV prevalence at a single point in time across the countries included in this study.

Generally, our findings on the changes by age group show that among younger women, there were declines in reported lifetime and current prevalence of violence across time points in India, Pakistan (physical violence) and Vietnam. However, there were increases in Timor-Leste (across all age groups) and in Nepal (among adolescent girls), and in the Philippines prevalence of current violence remained static across the three time points for the youngest age groups, while it declined among women aged 25 years or more. These findings highlights the vulnerability adolescent girls and young women face in intimate relationships in some settings, and that this age is a critical intervention group for violence prevention [5, 24–27]. In the context of increasing secondary school enrolment rates across the Asia Region, schools-based prevention programmes focused on developing healthy relationships could be a potential avenue to target this age group.

In both Timor-Leste and in the Philippines, there were notable increases in the percentage of women in cohabiting relationships. Social theories suggest that cohabiting relationships may be more prone to violence because of less commitment to the relationship [28], an assertion which has broader empirical support [29]. While in the Philippines the prevalence of both lifetime and current violence was higher among cohabiting women, prevalence, nevertheless, continued to steadily decline to a significant degree, highlighting that reductions in violence are also achievable in this group.

While the limitation of too few times points has been highlighted, the findings do suggest that awareness of violence against women is an important intervention point across the life-course, and health providers may be an important intervention point. In future, when data at more time points becomes available, ioinpoint regression analysis may be useful to identify significant trends in IPV prevalence over time. Additional limitations of this study include the use of indicators to measure sexual violence that are not consistent over different time points within countries. While it is possible that these differences have impacted the measured prevalence, the variation in indicators used in this study is slight. Furthermore, the focus on national estimates masks variation within countries, with evidence showing the importance of understanding sub-national nuances to develop effective and targeted policies and programs [30]. Finally, while the studies included in this analysis applied the same methodology within countries, it is important to stress that the findings reflect what women and girls were willing to disclose to the interviewers and that comfort to reveal personal experiences may also change over time [29]. Despite these limitations, the strengths of this analysis are the comparability of studies within countries because of the focus on exploring changes where the same methodology has been applied, and the large sample sizes of the studies reviewed which enable these changes to be demonstrated.

## Conclusion

This study sought to describe differences and changes in the prevalence of partner violence. By teasing out the relationship between women’s experiences of the different types of violence, severity of violence, and age changes, we contribute to a deeper understanding of women’s lived experiences in the region. Despite this, there are limitations in using survey data to explain change. If we are to reduce and prevent VAW globally there is a need for multiple time points and contextual analysis making use of information collected by other disciplines to achieve a deeper understanding of what is perceived to be driving or preventing change. Only when the hidden nuances are described and understood, will it be possible to truly develop evidence informed appropriate context specific policies and interventions.

## Data Availability

The datasets generated and/or analysed during the current study are available in the Macro DHS program repository, available from: http://dhsprogram.com/data/available-datasets.cfm.

## References

[1] UN Women. Action on ending violence against young women and girls. https://www.unwomen.org/en/what-we-do/youth/action-on-ending-violence-against-young-women-and-girls. Accessed 26 December 2020.

[2] WHO (2021). Violence against women prevalence estimates, 2018: Global, regional and national prevalence estimates for intimate partner violence against women and global and regional prevalence estimates for non-partner sexual violence against women.

[3] Campbell JC (2002). Health consequences of intimate partner violence. The Lancet.

[4] Ellsberg M, Jansen HA, Heise A, Watts CH, Garcia-Moreno C (2008). Intimate partner violence and women’s physical and mental health in the WHO multi-country study on women’s health and domestic violence: an observational study. The Lancet.

[5] Vyas S, Meinhart M, Troy K, Brumbaum H, Poulton C, Stark L (2021). The economic cost of violence against women and girls in low- and middle-income countries: a systematic review of the evidence. Trauma Violence Abuse.

[6] SDG. Goal 5- Achieve gender equality and empower all women and girls. https://www.un.org/sustainabledevelopment/gender-equality/. Accessed 25 December 2020.

[7] United Nations Population Fund (UNFPA). Violence against women – regional snapshot. https://asiapacific.unfpa.org/en/resources/violence-against-women-regional-snapshot-2020-knowvawdata. Accessed 24 March 2021.

[8] Garcia-Moreno C, Jansen HAFM, Ellsberg M, Heise L, Watts C. WHO Multi-country Study on Women’s Health and Domestic Violence against Women. Initial results on prevalence, health outcomes and women’s responses. Geneva: World Health Organization; 2005.

[9] Jansen, H.A.F.M. Measuring Prevalence of Violence Against Women: Survey Methodologies. UNFPA Asia; 2016. < https://asiapacific.unfpa.org/sites/default/files/pub-pdf/kNOwVAWdata%20Methodology.pdf>. Accessed 12 May 2023.

[10] DHS. Home page. https://dhsprogram.com/. Accessed 26 December 2020.

[11] WHO (2001). Putting women first: ethical and safety recommendations for research on domestic violence against women.

[12] Ellsberg M, Heise L (2005). Researching violence against women: a practical guide for researchers and activists.

[13] DHS. ‘Domestic Violence Module: Model Household Questionnaire.’ *The DHP Progra*, 2021. < https://dhsprogram.com/pubs/pdf/DHSQM/DHS8-Module-DomViol-Qnnaire-EN-12Nov2021-DHSQM.pdf>. Accessed 12 May 2023.

[14] Bott S, Guedes A, Ruiz-Celis AP, Mendoza JA. Intimate partner violence in the Americas: a systematic review and reanalysis of national prevalence estimates. Rev Panam Salud Publica. 2019;43. 10.26633/RPSP.2019.26.10.26633/RPSP.2019.26PMC642598931093250

[15] GSO (2010). Keeping silence is dying’: results from the national study on domestic violence against women in Viet Nam.

[16] MMOLISA, GSO, UNFPA (2020). Results of the national study on violence against women. Viet Nam 2019 - journey for change.

[17] Ackerson LK, Kawachi I, Barbeau EM, Subramanian SV. Effects of individual and proximate educational context on intimate partner violence: a population-based study of women in India. Am J Public Health. 2008; 98:507–514. doi:10.2105/AJPH. 2007.113738.10.2105/AJPH.2007.113738PMC225359018235066

[18] Jansen HAFM, Nguyen T, Hoang T (2016). Exploring risk factors associated with intimate partner violence in Vietnam: results from a cross-sectional national survey. Int J Public Health.

[19] Vyas S, Watts C (2009). How does economic empowerment affect women’s risk of intimate partner violence in low and middle income country settings?: a systematic review of published evidence. J Int Dev.

[20] Brown LJ, Lowe H, Gibbs A, Smith C, Mannell J (2022). High-risk contexts for violence against women: using latent class analysis to understand structural and contextual drivers of imtimate partner violence at the national level. J Interpers Violence.

[21] Fonseka RW, McDougal L, Raj A, Reed E et al. A mediation analysis of the role of girl child marriage in the relationship between proximity to conflict and past-year intimate partner violence in post-conflict Sri Lanka. Confl Health.2022; 16(5):1–12. 10.1186/s13031-022-00436-2.10.1186/s13031-022-00436-2PMC884281435164806

[22] Epstein, A., Bendavid, E., Nash, D., Edwin, D.,. Drought and intimate partner violence towards women in 19 countries in sub-Saharan Africa during 2011–2018: A population-based study. PLos Med. 2020;17(3). doi10.1371/journal.10.1371/journal.pmed.1003064PMC708198432191701

[23] Rao, S. A natural disaster and intimate partner violence: Evidence over time. Soc Sci Med. 2020; 247: 1–10. 10.1016/j.socscimed.2020.112804.10.1016/j.socscimed.2020.11280431978704

[24] Glass N, Fredland N, Campbell J, Yonas M, Sharps P, Kub J. Adolescent dating violence: prevalence, risk factors, health outcomes, and implications for clinical practice. J ObstetGynecol Neonatal Nurs. 2003;32:227–38. 10.1177/0884217503252033.10.1177/088421750325203312685675

[25] Raj A, Saggurti N, Lawrence D, Balaiah D, Silverman JG (2010). Association between adolescent marriage and marital violence among young adult women in India. Int J Gynaecol Obstet.

[26] Decker MR, Latimore AD, Yasutake S, Haviland M, Ahmed S, Blum RW, Sonenstein F, Astone AM (2015). Gender-based violence against adolescent and young adult women in low- and middle-income countries. J Adolesc Health.

[27] Engel et al. #ustoo- bringing violence against adolescent girls into focus. *Submitted to BMJ*.

[28] DeMaris A, Benson ML, Fox GL, Hill T, Van Wyk J (2003). Distal and proximal factors in domestic violence: a test of an integrated model. J Fam Stud.

[29] Abramsky T, Watts CH, Garcia-Moreno C, Devries K, Kiss L, Ellsberg M, Jansen HAFM, Heise L. What factors are associated with recent intimate partner violence? Findings from the WHO multi-country study on women’s health and domestic violence. BMC Public Health. 2011;11. 10.1186/1471-2458-11-109.10.1186/1471-2458-11-109PMC304914521324186

[30] Jansen H, Torres G, Yllo K (2020). Prevalence and patterns of sexual violence in marriage in the Pacific region: quantitative data in cross cultural comparison. Sexual violence in intimacy: implications for research and policy in global health.

